# Age-Dependent Decrease and Alternative Splicing of Methionine Synthase mRNA in Human Cerebral Cortex and an Accelerated Decrease in Autism

**DOI:** 10.1371/journal.pone.0056927

**Published:** 2013-02-20

**Authors:** Christina R. Muratore, Nathaniel W. Hodgson, Malav S. Trivedi, Hamid M. Abdolmaleky, Antonio M. Persico, Carla Lintas, Suzanne De La Monte, Richard C. Deth

**Affiliations:** 1 Department of Pharmaceutical Sciences, School of Pharmacy, Northeastern University, Boston, Massachusetts, United States of America; 2 Genetics Program, School of Medicine, Boston University, Boston, Massachusetts, United States of America; 3 Laboratory of Molecular Psychiatry and Neurogenetics, University Campus Bio-Medico, Rome, Italy; 4 Department of Medicine and Pathology, Rhode Island Hospital and Warren Alpert School of Medicine at Brown University, Providence, Rhode Island, United States of America; University of Sydney, Australia

## Abstract

The folate and vitamin B12-dependent enzyme methionine synthase (MS) is highly sensitive to cellular oxidative status, and lower MS activity increases production of the antioxidant glutathione, while simultaneously decreasing more than 200 methylation reactions, broadly affecting metabolic activity. MS mRNA levels in postmortem human cortex from subjects across the lifespan were measured and a dramatic progressive biphasic decrease of more than 400-fold from 28 weeks of gestation to 84 years was observed. Further analysis revealed alternative splicing of MS mRNA, including deletion of folate-binding domain exons and age-dependent deletion of exons from the cap domain, which protects vitamin B12 (cobalamin) from oxidation. Although three species of MS were evident at the protein level, corresponding to full-length and alternatively spliced mRNA transcripts, decreasing mRNA levels across the lifespan were not associated with significant changes in MS protein or methionine levels. MS mRNA levels were significantly lower in autistic subjects, especially at younger ages, and this decrease was replicated in cultured human neuronal cells by treatment with TNF-α, whose CSF levels are elevated in autism. These novel findings suggest that rather than serving as a housekeeping enzyme, MS has a broad and dynamic role in coordinating metabolism in the brain during development and aging. Factors adversely affecting MS activity, such as oxidative stress, can be a source of risk for neurological disorders across the lifespan via their impact on methylation reactions, including epigenetic regulation of gene expression.

## Introduction

Methionine synthase (MS) is a multi-domain enzyme which converts homocysteine (HCY) to methionine, utilizing methyl groups provided by 5-methyltetrahydrofolate (methylfolate) via a methylcobalamin (MeCbl) intermediate [1]–[4]. As illustrated in Fig. 1, HCY is formed as part of the methionine cycle of methylation via reversible hydrolysis of S-adenosylhomocysteine (SAH), which is in turn formed by methyl transfer from S-adenosylmethionine (SAM) in more than 200 different methylation reactions. MS activity also determines the level of tetrahydrofolate available for purine and thymidine synthesis. Furthermore, MS activity provides folate-derived methyl groups to the D4 dopamine receptor, supporting its unique ability to carry out dopamine-stimulated phospholipid methylation [5]–[7]. Thus MS activity influences an exceptionally wide range of cellular processes, thereby modulating metabolic activity in response to redox status.

**Figure 1:** Redox and methylation-related pathways in neurons. Neurons can utilize either astrocyte-derived or transsulfuration-derived cysteine for GSH synthesis; however, higher levels of cystathionine in human brain indicate impaired transsulfuration, increasing the importance of the former cellular uptake pathway. GSH levels are a primary determinant of cellular redox status, and oxidative stress can inhibit MS activity by multiple mechanisms, as described herein, including oxidation of Cbl(I), down-regulation of transcription, or alternative mRNA splicing with deletion of the cap domain. Oxidative stress restricts dopamine-stimulated phospholipid methylation, since it is dependent upon MS activity.

A decrease in MS activity counteracts oxidative stress by redirecting HCY to cysteine via the intermediate cystathionine. In most tissues, this transsulfuration pathway provides an important source of cysteine for glutathione (GSH) synthesis, but in brain transsulfuration activity is restricted by low activity of cystathionine-γ-lyase [8], although it still contributes to GSH synthesis [9]. Notably, the cystathionine level in human cortex is remarkably higher (∼40-fold) than in other human tissues, and a comparison of levels among other species revealed an evolutionary trend toward higher cystathionine [10], suggesting brain-specific regulation.

MS is composed of five structural domains, sequentially represented within its gene and mRNA, including HCY-binding, methylfolate-binding, cap, cobalamin-binding and SAM-binding domains [1]–[4] (Fig. 2). During the catalytic cycle, methylfolate-derived methyl groups are first transferred to the vitamin B12 co-factor (cobalamin) and then to HCY. The resulting Cbl(I) state of cobalamin is a highly reactive “supernucleophile”, which functions as a sensor/indicator of the cellular redox environment until it is again methylated [11]. However, during this vulnerable interval, the cap domain assumes a position above Cbl(I), partially protecting it from oxidation [2]. Cobalamin oxidation halts enzyme activity and diverts HCY to transsulfuration, which in turn, increases GSH synthesis until SAM-dependent reductive methylation of cobalamin restores MS activity [12]. This creates a negative feedback loop in which MS activity is sensitive to redox status and redox status is sensitive to MS activity.

**Figure 2:** Domain structure and exon composition of cobalamin-dependent MS. (**A**) MS is comprised of five domains: HCY-binding (pink), methylfolate-binding (green), cap (yellow), cobalamin-binding (red) and SAM-binding (blue). Structures from *E.coli* [1]–[3] and *T.maritima* [4] (PDB codes 1Q8J, 1K98 and 1MSK, respectively were used to construct a composite model). A structurally uncharacterized linker segment between the folate and cap domains is absent. (**B**) The human MS gene contains 33 exons specifying its five domains in a sequential manner. The location of PCR sequences used in this study is indicated by red and black line segments below the corresponding domains.

Many theories have linked aging to oxidation and increased mitochondrial production of reactive oxygen species (ROS) [13]–[15], which correspondingly increases the demand for antioxidant resources. However, the mechanism(s) by which cells adapt to this increasing demand have not been fully elucidated. Methylation of DNA and histones provides epigenetic regulation of gene transcription, which can be considered a candidate mechanism for adaptation to oxidative stress. Abnormalities affecting DNA methylation have been identified as primary causative factors for neurodevelopmental disorders such as Fragile-X, Rett, Angelman and Prader-Willi syndromes [16]–[20], and evidence of oxidative stress with impaired methylation has been frequently reported in autism [21]–[31]. Abnormalities within redox and methylation pathways are also linked to schizophrenia [32]–[38], Alzheimer's Disease (AD) [39]–[47], depression [48], [49] and other neuropsychiatric and neurological disorders [50], [51], suggesting a fundamental role in brain function.

While MS has commonly been regarded as a housekeeping enzyme, the above observations led us to hypothesize a unique role in human brain to regulate metabolism in response to redox status. We further hypothesized that MS status might be altered during aging and in neurological disorders associated with oxidative stress. To test these hypotheses we evaluated MS mRNA status in human frontal cortex and identified novel alternatively spliced transcripts. The level of MS mRNA displayed a remarkable age-dependent decrease, although protein levels of MS remained stable. While MS mRNA levels were lower in autistic subjects, protein levels were similar to control. Together our findings suggest a role for MS in coordinating transcription, translation and protein turnover across the lifespan in proportion to redox status, and disruption of this role in autism.

## Results

### Age-dependent changes in MS mRNA in human cortex

To investigate the status of MS mRNA in human cortex, PCR was used to probe cDNA libraries prepared from postmortem human cortex, obtained from Brodmann areas 22, 41, 42, or 46 (n = 47). In an initial study, PCR primers directed against each of the five domains of MS (Fig. 2B) were used to probe cortex-derived RNA from 24 year-old and 80 year-old subjects. Although the expected PCR products for all five domains were visualized for the 24 year-old subject (Fig. 3A), the cap domain product was absent for the 80 year-old subject (Fig. 3B). Additionally, a smaller size cap domain product in the 24 year-old sample suggested the possibility of alternative splicing.

**Figure 3:** MS mRNA in human cortex across the lifespan. Domain-specific PCR products for MS mRNA from 24 year-old (**A**) and 80 year-old (**B**) subjects. The predicted size of the PCR product is shown below each domain. Age-dependent decline in levels of MS mRNA was determined with (**C**) cobalamin-binding domain (**D**) or cap domain qRT-PCR primers. Data was fit to a two-component exponential function. (**E**) Cobalamin-binding and cap domain PCR products for subjects at 4, 49 and 84 years of age. GAPDH product for each pair of samples is show below. (**F**) Ratio of cap to cobalamin-binding qRT-PCR products for subjects <20 years *vs.* >60 years. ^*^ indicates significant difference from under 20 years group (p<0.0001).

To further explore the status of MS mRNA in postmortem human cortex, qRT-PCR was utilized to evaluate the level of cobalamin-binding and cap domain exons in subjects (n = 47) across the lifespan (28 weeks of fetal gestation to 84 years). For these studies cobalamin domain primers spanned exons 24 and 25, while cap domain primers spanned exons 19 and 20. A striking age-dependent decrease in mRNA levels was observed for both cobalamin and cap domains (Table 1; Figs. 3C and 3D). The decrease from fetal to >80 years of age amounted to ∼400-fold and ∼3,300-fold for cobalamin and cap domains, respectively. qRT-PCR data was best fit to a two-component exponential decay function, yielding fast and slow phase T_1/2_ values of 2.1 and 33.2 years (R^2^ = 0.90) and 2.1 and 23.5 years (R^2^ = 0.93) for cobalamin and cap domains, respectively. This pattern may reflect a progressive decrease in transcription and/or enhanced mRNA degradation. The age-dependent decrease is entirely attributable to a decrease in MS transcripts, since the level of GAPDH expression, which was used for normalization, was not significantly different for individuals <20 years *vs.* >65 years (p = 0.265) (data not shown). The decline in cobalamin and cap domain PCR products for representative samples is illustrated in Fig. 3E, whereas the level of GAPDH for each sample was unchanged.

**Table 1:** Control subject clinical details and CAP and COB mRNA values.

Case no.	Sex	Age (yrs)	PMI (hrs)	Cause of death	CAP mRNA A.U.	COB mRNA A.U.
A1	F	28 (wks)	Unknown	Unknown	634.57	564.03
UMB-1185	M	4	17	Drowning	296.11	315.36
UMB-1377	F	6	20	Drowning	205.07	205.42
UMB-1500	M	7	18	Multiple injuries	178.56	119.04
UMB-1860	M	8	5	Cardiac arrhythmia	166.57	149.87
UMB-1706	F	8	29	Rejection of heart transplant	97.68	95.32
UMB-1407	F	9	20	Asthma	121.94	128.25
B-6207	M	16	26	Ischemic heart attack	85.04	82.18
B-5251	M	19	18.6	Unknown	179.77	172.83
UMB-1541	F	20	19	Head injuries	146.02	188.95
B-3829	M	22	12	Central hepatic laceration	104.69	94.89
B-6221	M	22	24	Unknown	74.54	95.36
B-5718	M	22	21.5	Unknown	107.09	101.29
B-5601	M	24	21.3	Myocardial infarction	84.38	114.96
B-5873	M	28	23	Unknown	104.3	94.2
B-4211	M	30	23	Cardiac arrhythmia	50.56	55.20
B91	M	31	22	Cardiac arrest	61.64	32.46
B95	M	31	11	Pulmonary embolism	17.16	60.13
B-5352	M	31	33	Asphyxia	15.36	26.39
B83	M	32	13	Cardiac	9.79	40.17
B-6316	F	32	28.9	Unknown	77.05	72.07
B77	F	33	29	Asthma	17.89	63.96
B43	M	35	52	Myocarditis	7.34	6.30
B27	M	37	13	Cardiac arrest	4.27	4.57
B35	F	38	28	Cardiac arrest	10.90	13.56
B99	F	39	58	Cardiac arrest	21.42	57.81
B105	F	41	50	Cardiac arrest	78.29	56.72
B-5813	M	41	27.2	Unknown	51.54	71.51
B86	M	46	31	Cardiac arrest	18.01	20.69
B84	M	47	11	Cardiac arrest	17.22	12.65
B51	M	47	21	Cardiac arrest	28.46	10.97
B96	M	48	24	Cardiac arrest	31.36	27.11
B79	M	48	31	Cardiac arrest	8.73	15.36
B19	M	49	46	Cardiac arrest	12.39	13.14
B65	M	49	23	Cardiac arrest	6.07	10.06
B91	M	51	22	Cardiac arrest	30.82	10.56
B29	M	51	31	Cardiac arrest	17.28	18.52
B24	M	53	9	Cardiac arrest	28.26	30.71
B30	M	53	28	Cardiac arrest	9.82	13.32
B70	M	55	31	Cardiac arrest	14.78	13.89
B1L	F	57	9	Unknown	0.08	0.86
B38	M	60	47	Cardiac arrest	16.18	5.45
B1A	M	66.5	1	Unknown	0.01	0.31
B1D	F	72	3	Unknown	0.32	6.44
B1B	F	77.7	1.58	Unknown	0.04	0.70
B1F	M	80.8	4.25	Unknown	0.10	0.76
B1J	M	81.4	7.23	Unknown	0.22	1.95
B1C	M	83.7	2	Unknown	0.24	1.53

Control cortex samples from age 28 weeks to 84.7 years. A.U. = arbitrary units. PMI = postmortem interval.

Our cohort included 13 female and 34 male subjects. While a gender-based comparison using all subjects yielded no significant difference in the parameters for age-dependent decline, analysis of 10 age-matched pairs resulted in T_1/2_ values of 19.2 and 10.8 years for females and males, respectively, for a single-component exponential function. The difference between these values was significant (*p*<0.05), which suggests a possible gender-based difference in the rate of MS mRNA decline; however, the strength of this observation is limited due to the small number of female samples. Additionally, it is notable, but understandable, that accidental death was more common for younger subjects while cardiac arrest was more common for subjects older than 37 years, which could contribute to the pattern of age-dependent decrease in MS mRNA. However, the biphasic pattern of decrease is already evident for subjects <37 years.

The level of cap and cobalamin domain amplicons was compared for subjects ≤20 years *vs.* >60 years, yielding average values of 202.1±45.4 *vs.* 1.95±0.93 for cobalamin domain and 211.1±50.7 *vs.* 0.155±0.05 for cap domain. The resultant cap/cobalamin ratios of 1.045 and 0.079 were significantly different (*p*<0.0001) (Fig. 3F), indicating a greater age-dependent decrease in cap domain, as compared to cobalamin domain. Specifically, the more than 10-fold lower levels of cap domain in subjects >60 years indicates age-dependent alternative splicing of MS pre-mRNA which results in the loss of cap domain exons, and in turn, would account for the apparent absence of cap domain PCR product in the 80 year-old subject, as illustrated in Fig. 3A.

An examination of MS cDNA sequences deposited in the NCBI database revealed two examples of exon-skipping (accession numbers: AK299904.1 and BC144095.1). Exons 16–18 of the folate domain were deleted in a genome-wide study using a sample derived from fetal brain (accession number AK299904.1) [52] and exon 20 was deleted in a cDNA sequence derived from pooled human tissues which included cerebellum (accession number BC144095.1; age not specified) [53]. To further investigate alternative splicing, high-fidelity standard PCR was performed utilizing primers in exons 13 and 28, followed by gel separation and sequencing of the PCR products, for frontal cortex samples from a 20 week-old fetus and a 76 year-old subject. For both samples, three PCR products were identified, with the largest and most intensely stained band corresponding to the predicted full-length product (Fig. 4A), as confirmed by sequencing. The intermediate band was lower in intensity, and sequencing revealed that it lacked exons 16–18, coding for the C-terminal portion of the folate-binding domain. The lower band was consistently observed, but yielded too little material for sequencing. However, based upon its smaller size and the previous report of alternative splicing with exclusion of exons 19 and 20, these findings suggest that the lower size band lacks exons 16–20 (Fig. 4B). Together these three independent observations confirm the occurrence of multiple mRNA splice variants which involve deletion of portions of the folate-binding and cap domains of MS in human cortex.

**Figure 4:** MS mRNA variants in human cortex. (**A**) qRT-PCR was performed using cDNA from the cortex of fetal and 76 year old subjects, with primers spanning exons 13–26, yielding three products (a–c). (**B**) Exon composition of the full-length upper band (a) and the alternatively spliced middle band lacking exons 16–18 (b) were confirmed by sequencing; the proposed composition of the lower band is also illustrated (c).

### MS mRNA status in autism

Plasma levels of GSH are abnormally low in autistic children [21]–[25], and are generally observed in conjunction with higher levels of oxidative stress and inflammation biomarkers [26]–[29], while lower levels of SAM and higher levels of SAH are indicative of impaired MS activity [21], [22]. Moreover, levels of inflammation-associated cytokines such as tumor necrosis factor-alpha (TNF-α) are significantly elevated in CSF and postmortem brain samples from autistic subjects [30], [31], [54], which suggests that cortical MS status might be altered by oxidative stress in autism. To test this hypothesis, MS mRNA was evaluated by qRT-PCR in post-mortem cortical samples (Brodmann areas 9, 22, 41, 42 and 44) from age- and sex-matched autistic and non-autistic subjects ranging in age from 4 to 39 years (Table 2). Cobalamin and cap values for different Brodmann areas were not significantly different for either control or autistic subjects. Using primers directed against cobalamin-binding and cap domains, grouped data demonstrated that mRNA levels for both domains were significantly lower in autistic subjects than controls (*p*<0.01 for cobalamin domain; *p*<0.003 for cap domain), indicating reduced transcription of the MS gene (Fig. 5A).

**Figure 5:** Status of human cortex MS mRNA in autism. (**A**) Levels of cobalamin-binding (Cob) and cap domain (Cap) mRNA in grouped control *vs.* autistic subjects. * and ** indicate significant decreases compared to control group (*p* = 0.01 and 0.003, respectively). (**B**) Cobalamin-binding domain PCR products for age-paired control (C) and autistic (A) subjects. Age-pairs were 5 and 4 years, 11 and 9 years and 30 years. (**C**) Age-dependent levels of cobalamin-binding domain mRNA. Control data was best fit to an exponential decay function (T_1/2_ = 2.3 years; R^2^ = .97); Autism data was best fit to a linear function with slope not significantly different from zero. (**D**) Age-dependent levels of cap domain mRNA. Control data was best fit to an exponential decay function (T_1/2_ = 2.7 years; R^2^ = .94). Autism data was best fit to a linear function with slope not significantly different from zero. (**E**) Pair-wise comparison of cobalamin-binding domain mRNA for different autism age groups. (**F**) Pair-wise comparison of cap domain mRNA for different autism age groups.

**Table 2:** Control and autistic subject clinical details and CAP and COB mRNA values.

Case no.^a^	Sex	Age (yrs)^b^	PMI (hrs)^c^	Brodmann Area	Cause of death	CAP mRNA A.U.	COB mRNA A.U.
**Controls:**							
UMB-1185	M	4	17	9	Drowning	296.11	315.36
UMB-1377	F	6	20	9	Drowning	205.07	205.42
UMB-1500	M	7	18	41/42	Multiple injuries	178.56	19.04
UMB-1860	M	8	5	45	Cardiac arrhythmia	166.57	149.87
UMB-1407	F	9	20	22	Asthma	121.94	128.25
B-6207	M	16	26	9	Ischemic heart attack	85.04	82.18
UMB-1541	F	20	19	41/42	Head injuries	146.02	188.95
B-3829	M	22	12	9	Central hepatic laceration	104.69	94.89
B-5718	M	22	21.5	41/42	Unknown	107.09	101.29
B-6221	M	22	24	45	Unknown	74.54	95.36
B-5601	M	24	21.3	41/42	Multiple injuries	84.38	114.96
B-5873	M	28	23	41/42	Unknown	104.3	94.2
B-4211	M	30	23	22	Cardiac arrhythmia	50.56	55.20
B-5352	M	31	33	41/42	Asphyxia	15.36	26.39
B-6316	F	32	28.9	41/42	Unknown	77.05	72.07
B-5813	M	41	27.2	41/42	Unknown	51.54	71.51
**Autism:**							
UMB-4671	F	4	13	9	Accident	28.64	33.12
B-5569	M	5	25.5	9	Drowning	88.65	84.45
UMB-1349	M	5	39	44	Drowning	119.24	111.28
B-7002	F	5	32.7	41/42	Drowning	98.3	87.8
UMB-4721	M	8	16	9	Drowning	91.14	71.51
B-5666 †	M	8	22.2	41/42	Unknown	55.33	94.07
B-1182	F	9	24	41/42	Smoke inhalation	46.88	37.97
B-4925	M	9	27	41/42	Seizure disorder	39.42	34.52
*UMB-144*†	M	10	22	22	Drowning	63.12	59.91
B-5342	F	11	13	9	Drowning	76.64	99.73
B-6294	M	16	Unknown	44	Unknown	95.67	117.03
B-5144	M	20	23.7	44	Traffic accident	68.12	62.74
B-6677	M	20	16	41/42	Congestive heart failure	54.22	32.6
B-1638	F	21	50	41/42	Respiratory failure during S.E.	44.97	38.27
B-6337	M	22	25	9	Choking	42.22	43.71
B-5000	M	27	8.3	41/42	Drowning	13.98	60.58
B-6640	F	29	17.8	41/42	Seizures	0.61	1.46
B-6994	M	29	43.2	22	Seizures	5.34	13.94
B-5173	M	30	20	9	Gastrointestinal hemorrhage	58.49	38.36
B-6401	M	39	14	41/42	Cardiac tamponade	32.46	38.83

a Autism Tissue Program identifier. All autistic samples were paired with age- and sex-matched controls.

b Mean age (± s.d.) for control group = 20.1±6.6, for autism = 16.4±10.4; paired-t = 1.055, df = 34, *P* = 0.299.

c Mean PMI (post-mortem interval) (± s.d.) for control group = 21.2±6.6, for autism = 23.8±10.9; paired-t = 0.8428, df = 33, *P* = 0.405. Statistical results indicate no mean differences in age or PMI. † Autism samples that were not pair-matched, but included in the mean MS mRNA analysis. *Italics* indicate cases of PDD-NOS (Pervasive Developmental Disorder Not Otherwise Specified). A.U. = arbitrary units. S.E. = status epilepticus.

While control subjects displayed an age-dependent decrease in MS mRNA levels across the 4 to 42 year interval, this was not the case for autistic subjects (Fig. 5B-D). Control subject data, for cobalamin and cap domains, was best fit to a one-component exponential function, yielding T_1/2_ values of 2.3 years (R^2^ = 0.97) and 2.7 years (R^2^ = 0.94), respectively. However, autism subject data was best fit by a straight line with a slope not significantly different from zero, which indicates the absence of an age-dependent decrease during this interval. The autism-associated decrease in mRNA was similar for both cobalamin (48%) and cap (50%) domain primers, indicating that the total number of MS transcripts was reduced, as opposed to a change in alternative splicing. A pair-wise comparison confirmed that the amount of decrease in MS mRNA was greatest for younger autistic subjects, when levels are normally higher (Figs. 5E and F). The difference between paired samples followed an exponential decline with age, yielding T_1/2_ values of 1.8 and 2.7 years for cobalamin and cap domains, respectively, corresponding to an absence of the early phase of rapid MS mRNA decline. While the limited number of samples means that our findings are clearly preliminary, our data suggests that autism is associated with prematurely low levels of MS mRNA in cerebral cortex.

### MS protein levels

Due to the age-dependent decrease and alternative splicing of MS mRNA transcripts, immunoprecipitation and western blotting were used to examine MS protein status in postmortem cortex samples. An antibody directed against the N-terminal HCY-binding domain detected three major protein bands with approximate MWs of ∼140, 113 and 101 kDa. The most abundant form of MS was the 101 kDa splice variant, which was greater than the 140 or 113 kDa bands (Fig. 6A). Full-length MS has a predicted MW of 140.5 kDa and exons 16–18 would contribute 16.4 kDa, while exons 16–20 would contribute 25.5 kDa. Therefore, the ∼10 kDa difference between the two lower MW protein species roughly corresponds to presence or absence of exons 19 and 20, but the apparent MW values of the two variant protein forms are lower than expected from mRNA splice variants. This might indicate additional deleted exons beyond those characterized in this study or unblocked proteolysis. Surprisingly, despite significant differences in mRNA levels, levels of MS protein were not different between young *vs.* old subjects or autistic *vs.* control subjects, and each group displayed similar levels of the three variants (Fig. 6B). As discussed below, the age-dependent decrease in RNA to protein ratio may reflect a unique role for MS in coordinating transcription, translation and protein turnover.

**Figure 6:** MS protein status in human cortex. (**A**) Western blot analysis of MS protein revealed three primary bands with approximate MW values of 140, 113 and 101 kDa. A similar pattern was observed for young control subjects, age-matched autistic subjects, and elderly subjects. (**B**) Quantification of western blot data. The density of the three MS variants was not significantly different between the three groups (n = 8).

### Sulfur metabolite and redox status in autism

Lower MS mRNA in autistic subjects may be associated with an imbalance of the sulfur-containing metabolites involved in methylation, transsulfuration or antioxidant pathways. To examine this possibility, the levels of sulfur metabolites in postmortem cortical samples from control (n = 8) and autistic (n = 10) subjects were examined. Age and postmortem interval (PMI) for the two groups were not significantly different, and there was no significant relationship between any metabolite level and PMI. As illustrated in Fig. 7, a significant decrease in the levels of HCY and cystathionine was observed in autism samples (*p*<0.05), whereas levels of other metabolites were comparable between the two groups. The combined decrease in HCY and cystathionine suggests activation of the transsulfuration pathway, which supplies cysteine for GSH synthesis, especially during oxidative stress [55]. Levels of 8-OH guanosine, a biomarker of oxidative stress, were not significantly different between control and autistic subjects (0.65±0.11 and 0.67±0.06 ng/mg RNA, respectively).

**Figure 7:** Redox and methylation pathway metabolite levels in frontal cortex of autistic and control subjects. Tissue homogenates were prepared from autistic (n = 11) and control (n = 8) subjects and thiol/thioether metabolite levels were analyzed via HPLC with electrochemical detection. Levels of homocysteine and cystathionine were significantly lower in autistic subjects (*p*<0.05).

### TNF-α inhibits MS transcription

The pro-inflammatory cytokine TNF-α increases cystathionine-â-synthase activity and augments transsulfuration [56], and its levels are elevated in CSF and postmortem brain of autistic individuals [31], [54], as well as in amniotic fluid obtained during their fetal development [57]. To investigate whether inflammation might contribute to decreased levels of MS mRNA, cultured human SH-SY5Y neuroblastoma cells were treated with TNF-α (30 ng/ml), and levels of cobalamin and cap domain-containing transcripts were measured at different time intervals. As shown in Fig. 8A, TNF-α caused a prompt and substantial decrease in MS mRNA, reaching a >90% reduction after 45 minutes. Both cobalamin and cap domain transcripts were decreased, with the maximum decrease being somewhat greater for cobalamin *vs.* cap domain (80.3% *vs.* 64.4%).

**Figure 8:** TNF-α regulation of MS mRNA, cysteine uptake and thiol/thioether metabolites in SH-SY5Y human neuroblastoma cells. Confluent SH-SY5Y cells were treated with TNF-α (30 ng/ml) for the specified period of time, after which MS mRNA was analyzed via qRT-PCR (**A**), or cysteine uptake was measured (**B**) or cellular thiol and thioether metabolites were measured by HPLC with electrochemical detection (**C**). A significant decrease (*p*<0.05) in MS mRNA cobalamin domain mRNA transcripts was observed as early as 15 min and was sustained for 120 min (**A**). A significant decrease (*p*<0.05) in cysteine uptake was observed beginning at 20 min that was sustained for 240 min. (**B**). Time-dependent changes in redox/methylation metabolites included a transient increase in cysteine and GSH, as well as sustained decreases in methionine, cystathionine and homocysteine (**C**).

To further investigate the actions of TNF-α, its influence on cellular uptake of cysteine and the level of redox-related metabolites was also evaluated. TNF-α significantly decreased cysteine uptake, similar in time to its reduction of MS mRNA levels (Fig. 8B). Surprisingly, this decrease in uptake was not associated with a decrease in cellular cysteine levels. However, a significant increase was observed after 30 minutes, followed by a return to pretreatment levels (Fig. 8C). This transient increase was mirrored in changes of the GSH level, reflecting its cysteine dependence, while cystathionine and methionine levels decreased by >50% and HCY decreased to a modest extent. Together, these changes indicate that TNF-α promotes an increase in transsulfuration and a decrease in cysteine uptake, both of which are associated with and result in decreased MS transcription.

## Discussion

MS activity exerts a broad influence over cellular function by virtue of its involvement in four important metabolic pathways: transsulfuration, methylation, dopamine-stimulated phospholipid methylation and single-carbon folate pathways (Fig. 1). Vulnerability of its cobalamin cofactor to oxidation renders each of these pathways redox-sensitive [3], making MS an exceptional candidate for coordinating metabolic activity in response to changes in the oxidative environment. The current study demonstrates a dramatic age-dependent decrease of MS mRNA levels in human frontal cortex of almost 500-fold, accompanied by alternative splicing that results in three variant protein forms. Despite this remarkable decrease in MS mRNA, levels of MS protein were not changed across the lifespan. We also document lower MS mRNA levels and the absence of an age-dependent trend in autistic subjects. Together, these findings highlight a previously unappreciated complexity in MS regulation in frontal cortex during neurodevelopment, which is disrupted in autism.

### Redox-dependent methylation in brain

The threat of oxidative damage has been a critical driving force for evolution, and the emergence of cobalamin synthesis significantly influenced the evolutionary trajectory of metabolic networks [58]. Since human cortex reflects recent evolution, it may express unique redox-related metabolic features, as evidenced by a remarkable evolutionary trend for higher brain levels of cystathionine [10]. Additionally, cysteine and GSH levels in human CSF are more than 10-fold lower than plasma [59]. Coupled with a high rate of oxygen consumption, this scarcity of extracellular antioxidant resources makes the brain particularly vulnerable to oxidative insults and increases the need for adaptive responses to sustain sufficient intracellular GSH for neurons to survive 70+ years, while at the same time keeping them from dividing. Redox-dependent modulation of MS activity allows methylation reactions, including epigenetic regulation of gene expression, to participate in adaptive responses. Moreover, the activities of >200 SAM-dependent methyltransferase enzymes coded within the human genome are rendered redox-sensitive by cobalamin-dependent MS [60].

The levels of MS protein or mRNA in human brain across an entire lifespan were previously unknown. MS was included in a recent genome-wide study of transcription in human cortex [61], but unfortunately the primers utilized were targeted to the non-coding 3′ portion of the gene. We found a robust decrease in MS mRNA extending from fetal development through the end of adolescence, subsiding to a more gradual decrease during adulthood. Aging is associated with a decrease in plasma GSH and cysteine levels, while cystine and HCY levels increase [62]–[66]. CSF HCY levels in 17–40 *vs.* 69–86 year-old cohorts found an increase of 85% in the older cohort [67], indicative of decreased MS activity and consistent with the slow component of decreasing MS mRNA across this age range in our study (Fig. 3c and d).

Recent studies describe global patterns of changing gene expression and DNA methylation status in postmortem prefrontal cortex across the lifespan [61], [68]. Transcription of a large number of genes changed dramatically during the fetal to infant transition, primarily changing from high expression to low expression, and this pattern was reversed 50 years later, during aging and neurodegeneration [60]. Changes in DNA methylation were most dynamic during fetal development, becoming progressively smaller with age, and genes that were unmethylated during fetal development commonly became more methylated during the postnatal period [68]. The changes in MS mRNA levels we observed may be related to these global changes in DNA methylation and transcription.

### Implications for brain disorders

Oxidative stress and impaired methylation may be of etiologic importance in a number of neuropsychiatric and neurodegenerative disorders. The post-adolescent transition from a rapid decrease to a slow decrease in MS mRNA (Fig. 3) suggests an important transition in redox and methylation metabolism upon cessation of growth. This is a vulnerable period for the onset of schizophrenia, which has recently been linked to oxidative stress and low levels of GSH [34]–[38], while treatment with N-acetylcysteine, which augments GSH synthesis, has been shown to improve schizophrenia symptoms [69], [70]. The subsequent slow age-dependent decrease in MS mRNA may reflect further adaptation to oxidative stress, which is a risk factor for a number of neurodegenerative disorders [40], [41]. Notably, a SNP (A2756G) in the MS gene (MTR*)* has been linked to increased risk of sporadic AD [42]. Plasma levels of HCY are elevated in late-onset AD [71]–[73], and the rate of cognitive decline is correlated with HCY levels [74]. AD is associated with epigenetic drift, which in turn affects the methylation status of AD-risk genes, such as apolipoprotein E4 (APOE4) [45]. In support of this perspective, supplementation with vitamins B6 and B12 and folic acid is reported to significantly reduce the progression of AD neurodegeneration [75].

Since changing patterns of gene expression are intimately related to development, it is not surprising that disruption of DNA methylation is associated with genetic neurodevelopmental disorders such as Fragile-X, Rett, Angelman and Prader-Willi syndromes [16]–[20], as well as autism [76]–[78]. The lower level of MS mRNA in autistic subjects (Fig. 6) may be an adaptive response to abnormally increased antioxidant demand, with epigenetic and neurodevelopmental consequences. While ours is only a preliminary observation, this perspective is consistent with studies documenting oxidative stress and neuroinflammation in autistic children [21]–[31], [54], and reports of abnormal DNA methylation in autistic brain [76], [79], [80], including a study involving many of the same subjects as in this study, which demonstrated hypermethylation of the oxytocin receptor [80]. Recent postmortem studies document decreased GSH and increased oxidative stress in cerebellum and temporal cortex of autistic subjects [81], [82], although, similar to our results, GSH levels were not significantly lower in frontal cortex [81]. This may indicate region-specific differences in the ability to adapt to oxidative stress, and the decreased MS mRNA we observed in autistic subjects may reflect an oxidative stress-induced acceleration of the normal rate of decline. Genetic factors play an important role in autism, and single-nucleotide polymorphisms (SNPs) affecting MS activity have been documented to occur with higher frequency in autistic subjects [21], [24].

Elevated CSF TNF-α in autistic subjects [31] prompted our examination of a possible role for this proinflammatory cytokine in decreasing MS mRNA in autism. We observed a marked reduction in MS mRNA within an hour of TNF-α exposure, in SH-SY5Y neuroblastoma cells (Fig. 9). Thus it can be inferred that TNF-α-mediated inflammation is a candidate for causing lower levels of MS mRNA in autism. TNF-α promotes GSH synthesis by augmenting transsulfuration, in association with cleavage of a SAM-binding inhibitory domain in cystathionine-â-synthase [56], and decreased MS activity would further augment transsulfuration. Autistic individuals with elevated TNF-α would therefore be at greater risk of impaired methylation. The cause of elevated TNF-α in autism is unclear. However, elevated levels in amniotic fluid from mothers of children who developed autism [57] suggest the importance of prenatal or genetic factors.

**Figure 9:** Redox-dependent global metabolic regulation by MS. MS activity is highly sensitive to redox status and in turn affects redox status via its influence over transsulfuration of HCY to cystathionine and cysteine. TNF-α transcription is under the epigenetic control of methylation and exerts a potent negative influence over MS mRNA levels. Changes in MS activity affect >200 methylation reactions via the SAM to SAH ratio, grouping all these reactions under the influence of redox status. Methylation regulates fundamental aspects of metabolism, including gene expression RNA processing and protein turnover. The requirement of MET t-RNA for initiation of protein synthesis underscores the central role of MS in the global coordination of metabolism.

### MS and metabolic homeostasis

Alternative mRNA splicing allows formation of multiple protein products from a single gene, greatly increasing metabolic complexity and flexibility. Alternative splicing is particularly active in human brain [83], [84] and the current study highlights MS as an example. Three isoforms of MS at both protein and mRNA levels were identified: the full length enzyme, along with variant forms lacking exons 16–18 (missing the C-terminal portion of the folate-binding domain) or exons 16–20 (missing both the C-terminal folate-binding domain and the N-terminal portion of the cap domain). Deletion of exons 19 and 20 was particularly prominent in mRNA transcripts for subjects >60 years of age, but protein levels of the three MS variants remained constant throughout the lifespan. Deletion of exons 16–18 would be expected to decrease methylfolate-binding affinity, while deletion of exons 19 and 20 would be expected to increase vulnerability of Cbl(I) to oxidation, but further studies are needed to delineate the functional consequences of alternatively spliced forms of MS. We hypothesize that full-length MS has the lowest potential for oxidation, followed by the alternatively spliced form missing exons 16–18, while the alternatively spliced form missing exons 16–20 is most vulnerable to oxidation. Thus alternatively spliced forms of MS may increase its sensitivity to ROS, which in turn increases the responsiveness of methylation reactions to changes in cellular redox status.

The remarkable stability of MS protein levels across the lifespan, despite large changes in mRNA levels, reflects its central role in regulating and coordinating cellular metabolism at essentially every level, from genomic transcription to metabolite concentrations. As summarized in Fig. 9, MS exerts global epigenetic control over gene transcription through its influence over methylation of DNA and histones, while methylation of spliceosomal RNA [85], along with patterns of exon/intron DNA methylation [86], regulates alternative splicing. Nascent mRNA transcripts are methylated, particularly at their 5′-termini, which contributes to their stability [87]. Methylation of ribosomal RNA and tRNA regulates translation efficiency [88], and most critically, methionyl-tRNA is required for initiation of protein synthesis [89], ensuring that new protein synthesis will occur in proportion to availability of methionine. Protein degradation is also under the influence of methylation, since N-methylation of lysine residues interferes with ubiquitination, thereby prolonging protein lifespan [90]. Thus as protein lifespan increases, mRNA levels will decrease to maintain the same protein level and the same level of metabolites. The combined influence of MS on protein synthesis and degradation, coupled with its sensitivity to inactivation by ROS, enables global adjustment of cellular metabolism in proportion to redox status.

An association between TNF-α and aging has been extensively documented [91]. By simultaneously inhibiting MS transcription and augmenting CBS activity, TNF-α shifts the disposition of HCY away from methylation and toward transsulfuration, thereby increasing antioxidant synthesis in coordination with diminished methionine synthesis. Neuroinflammation and increased TNF-α during early brain development could accelerate the progressive age-dependent decrease in protein turnover, resulting in diminished neuroplasticity and learning capacity. Interestingly, restriction of dietary methionine increases longevity, in association with increased GSH levels [92] and increased transsulfuration, while rates of mRNA translation and protein levels are decreased [93], [94]. Auto-regulatory decreases in transcription, translation and protein turnover help sustain homeostatic equilibrium across the lifespan, and these adaptive changes represent signs of aging. Taken together, our results suggest an important role for MS in coordinating metabolic responses to redox changes during aging, elevating its status from that of a housekeeping enzyme to a central factor in maintaining redox equilibrium.

Our findings are subject to several important limitations. The overall number of brain samples was limited, and a larger study would provide a more accurate description of age-related and/or gender-related differences in MS mRNA status. More specifically, the relatively small number of autistic samples makes our observations preliminary in nature and subject to confirmation. Our studies were limited to MS status in frontal cortex and follow-up studies should evaluate lifespan-related changes in other brain regions as well as other tissues. Pairwise analysis of autistic and control samples from matched anatomical locations within frontal cortex would provide an important further test of our preliminary findings. We only investigated alternative splicing for a limited number of exons and a complete analysis of MS mRNA splicing might yield additional insights. The relative contribution of neurons *versus* glial cells to changes in MS mRNA was not addressed by our studies, which could be clarified by analysis of transcript density at the cellular level.

## Materials and Methods

### Tissue Samples

Postmortem human frontal cortex, RNA, and cDNA samples from autistic patients and control subjects (Brodmann areas 9, 22, 41, 42, or 46) were obtained through the Autism Tissue Program (ATP), the Australian Brain Bank Network (ABBN) and the Stanley Medical Research Institute (SMRI). A sample of fetal cortex RNA (28 weeks of gestation) was purchased from Invitrogen™. Control subjects ranged from 28 weeks to 83 years (n = 41), and their clinical details are provided in Table 1. Autistic subjects and their age-matched controls were ages 4 to 30 years (n = 10) (Table 2). Sample RNA was isolated using RNAqueous® -4PCR Kit from Ambion®. All samples were treated with DNase to remove trace DNA contamination. The project was conducted with the approval of the Institutional Review Board of Northeastern University.

### RT-PCR Amplification

cDNA synthesis and subsequent PCR amplification was performed using the Cloned AMV First-Strand cDNA Synthesis Kit and Platinum® Taq DNA Polymerase High Fidelity from Invitrogen™. cDNA synthesis used 1 ìg RNA and random oligo primers. RT-PCR was performed using 2 ìL of cDNA with 50 mM MgSO_4_ and 10 ìM sense and antisense primers; the primer annealing temperature used was 60°C.

### Quantitative Real-Time PCR (qRT-PCR)

Custom primers to each domain of human MS, as well as to exons 15–21, were designed and synthesized, as well as primers for GAPDH (Table 3). In the case of cap and cobalamin domains, different primer sets (Cap 2 and Cobalamin 2) were selected for qRT-PCR studies. qRT-PCR was performed on duplicate samples using the ABI Prism 7000 Sequence Detection System (Applied Biosystems™) under the following thermal cycling parameters: 2 min at 50°, followed by 10 min at 95°, and then 40 cycles of 95° for 15 sec, 60° for 1 min and 72° for 45 sec, followed by a final extension of 72° for 5 min. Values were normalized to GAPDH and data was analyzed using the ΔΔCt method [95].

**Table 3:** Primer Sequences.

Primer	Sequence 5′→ 3′	Amplicon Size (bp)
Homocysteine	ACATGTGCTCTGCAGGAGTG	187
	GCCTGCTCTTGGTATGCTTC	
Folate	TGGAGAGCGCTGTAATGTTG	197
	CTGGCTCGGAAGCAATTAAG	
Cap 1 (exons 19–21)	CGAAGAACGCCTTGAGTATGC	288
	TCTTCTACTGTGCCGTTAAGC	
Cap 2 (exons 19–20)	GGCACAGGAGGGAAGAAAGT	180
	TTCATCAGGGGTCCTTCAAT	
Cobalamin 1 (exons 22–23)	TGCACGACATAGGCAAGAAC	122
	TGCTTTGTGGTCAAGAGCAG	
Cobalamin 2 (exons 24–25)	CACTCCTTCCCTGGATGAAA	108
	TGCTGTGTGGGTTTTTGAAG	
S-Adenosylmethionine	AGGCCAGGAAGGTCTACGATG	300
	AGCAGGCAACGGCAAAC	
MS exons 15–21	ATGGAGCTGCTATGGTGGTC	847
	CCCTGGTAAGGGTCCTCTTC	
MS exons 13–28	TGGAGAGCGCTGTAATGTTG	1866
	ATCTTGGGAAAGCCTCGATT	
GAPDH	GAGTCAACGGATTTGGTCGT	238
	TTGATTTTGGAGGGATCTCG	

Primers are listed as forward and reverse for each set.

### Immunoprecipitation and Western Blot

A 10% homogenate of postmortem brain samples was prepared in lysis buffer and gently shaken at 4°C for 2 hours before centrifugation. 100 µl of the supernatant was incubated overnight at 4°C with 5 µl of rabbit-derived anti-MS antiserum followed by precipitation for 4 hours with protein A-coupled sepharose beads. After centrifugation and washing of the pellet, samples were size-fractionated by SDS-PAGE and the blot was transferred to Immobilon-PVDF membranes (Millipore). The blot was first incubated in blocking buffer (5% milk, 0.1% Tween in PBS) at room temperature for 1 hour and subsequently incubated with anti-MS antibody in precooled blocking buffer overnight at 4°C. After washing in PBS/0.1% Tween, blots were incubated with horseradish peroxidase (HRP)-labeled anti-rabbit secondary antibody at room temperature for 1 hour, after washing with PBS/0.1% Tween, developed by enhanced chemiluminescence (GE Healthcare Biosciences), and visualized with Hyperfilm-ECL (GE Healthcare Biosciences). Protein bands were quantified using TotalLab Quant® software (TotalLab).

### Thiol Metabolite Analysis

Thiol and thioether metabolites were measured using high performance liquid chromatography (HPLC) with electrochemical detection. Brain samples were thawed on ice, and a 10% homogenate was prepared. 50 µL of a 0.4 N perchloric acid solution was added to 200 ìL of the sample, and samples were gently blown with nitrogen gas before being centrifuged at 13,000 RPM for 60 min. A 100 ìL of sample was added to a microautosampler vial, blown with nitrogen gas, capped and loaded at 4°C in the ESA model 245 autosampler cooling tray. 10 ìL of sample was injected into a HPLC system via the autosampler. Metabolites were separated using an ESA dual pump HPLC system, pump model 584, Agilent Eclipse XDB-C8 (3×150 mm; 3.5 ìm) reverse-phase C8 column. A dual mobile phase gradient elution consisted of a mobile phase containing 25 mM sodium phosphate and 2.8 mM 1-octanesulfonic acid, adjusted to pH 2.65 with phosphoric acid, and a second mobile phase that was the same as the first, but additionally contained 50% acetonitrile. The system was run at a flow rate of 0.6 mL/min at ambient temperature with the following gradient: 0 to 9 min at 0% mobile phase B; 9 to19 min (50% B); and 19 to30 min (50% B). After each run, the column was re-equilibrated with 5% B for 12 minutes. Thiol and thioether metabolites were quantified using an ESA CoulArray with boron diamond-doped analytical cell model 5040 electrochemical detector operating at 1500 mV. Peak area analysis, based on standard curves generated for each compound, was performed using CoulArray software (version 3.06 ESA analysis program package).

### 8-Oxo-guanosine Analysis

To measure the state of oxidative RNA damage, 8-hydroxyguanosine (8-OHG) levels were quantified from RNA extracted from brain samples using the OxiSelect RNA damage enzyme-linked immunosorbent assay (ELISA) kit (Cell Biolabs, Inc, San Diego, CA), according to the protocol provided by the company.

### Cultured Cells Studies

SH-SY5Y human neuroblastoma cells from American Type Culture Collection were grown in α-MEM media supplemented with 10% (v/v) fetal bovine serum and 1% (v/v) penicillin-streptomycin-fungizone at 37° in a humidified 5% CO_2_-containing atmosphere. Prior to cysteine uptake or qRT-PCR studies or determination of cellular thiol levels, cells were treated with 30 ng/ml of TNFα for the indicated time periods.

### Cysteine Uptake Studies

Cells were grown to confluence in six-well plates and treated with 30 ng/ml of TNFα for the indicated period of time. Media was aspirated and cells were washed with Hank's balanced salt solution (HBSS). Non-radioactive HBSS was replaced with 600 µl of HBSS containing 10 µM [35S]-cysteine (1 µCi/ml) and 100 µM DTT, followed by a 5 min incubation. The [^35^S]-cysteine/HBSS mixture was aspirated and treatment was terminated with 2X washes of ice-cold HBSS. Cells were then lysed, scraped, and collected in a microcentrifuge tube, and then sonicated for 10 seconds. An aliquot of the sonicate was retained for protein estimation and the remainder counted for [^35^S] content. Cysteine uptake was expressed as nmoles/mg protein.
